# Diagnostic Value of Model-Based Iterative Algorithm in Tuberculous Pleural Effusion

This article has been retracted.

**DOI:** 10.1155/2022/7845767

**Published:** 2022-02-09

**Authors:** Suya Xi, Jinhao Sun, Hongjing Wang, Qingzhe Qiao, Xianghong He

**Affiliations:** ^1^Department of Respiratory and Critical Care Medicine, Hebei Chest Hospital, Shijiazhuang, Hebei 050000, China; ^2^Department 5 of Tuberculosis, Hebei Chest Hospital, Shijiazhuang, Hebei 050000, China; ^3^Second Department of Respiratory Medicine, Hebei Chest Hospital, Shijiazhuang, Hebei 050000, China; ^4^Department of Respiratory Medicine, Hebei Chest Hospital, Shijiazhuang, Hebei 050000, China

## Abstract

Although there are several diagnostic modalities for tuberculous pleurisy, there is still a lack of easy, cost-effective, and rapid methods for confirming the diagnosis. In order to facilitate clinicians to diagnose patients with tuberculous pleurisy at an early stage, help patients to obtain treatment early, and reduce lung damage, it is hoped that new techniques will be available in the future to help diagnose tuberculous pleurisy rapidly in the clinic. To this end, this paper investigates the problem of bidirectional consistency based on event-triggered iterative learning. Firstly, a dynamic linearized data model of TB pleurisy intelligent system is established using compact-form dynamic linearization method, and a parameter estimation algorithm of TB pleurisy data model is proposed; then, based on this data model, an output observer and a dead zone controller are designed, and an event-triggered distributed model-free iterative learning bidirectional consistency control strategy is constructed by combining with signal graph theory. In this paper, 112 patients with pleural effusion were collected, including 76 patients with confirmed or clinically diagnosed tuberculous pleural effusion and 36 patients with nontuberculous pleural effusion. Pleural effusion T-SPOT.TB, blood T-SPOT.TB, pleural effusion Xpert MTB/RIF, and pleural effusion adenosine deaminase (ADA) tests were performed before treatment in the included patients. The sensitivity of pleural effusion T-SPOT.TB was higher than that of peripheral blood T-SPOT.TB (76.32%, 58/76), pleural effusion Xpert MTB/RIF (65.79%, 50/76), and pleural effusion ADA (28.95%, 22/76); the differences were statistically significant (*x*^2^ = 14.74, 25.22, and 76.45, *P* < 0.01). The specificity of the Xpert MTB/RIF test for pleural effusion (100%, 36/36) was higher than that for pleural effusion T-SPOT.TB (77.78%, 28/36), peripheral blood T-SPOT.TB, and pleural effusion T-SPOT.TB. The sensitivity of the combined Xpert MTB/RIF test (64.47%, 49/76) was lower than that of the pleural effusion T-SPOT.TB alone (97.37%, 74/76).

## 1. Introduction

Our country is a high-burden country for pulmonary tuberculosis, and tuberculous pleurisy is included in the category of pulmonary tuberculosis [1]. The literature reports that tuberculous pleurisy is divided into dry pleurisy and exudative pleurisy, with dry pleurisy being an early inflammatory response of the pleura and exudative pleurisy presenting mainly as pleural effusion.

Pleural effusion in tuberculous pleurisy is the result of a combination of factors [2]. As the caseous lesions under the pleura break down, leading to the release of *Mycobacterium tuberculosis* antigens into the pleural cavity, the inflammatory response of the body's immune cells to anti-*Mycobacterium tuberculosis* antigens leads to increased capillary permeability, allowing plasma proteins to enter the pleural cavity, and the increased protein content in the pleural fluid stimulates the pleura to produce more pleural fluid; pleural inflammation leads to the formation and accumulation of pleural fluid due to the obstruction of the lymphatic vessels of the pleural wall layer by the involvement of pleural fluid reflux pleural fluid; neutrophils are mainly involved in the initial 24 h of the inflammatory response, macrophage numbers peak at 96 h after the onset of inflammation, and T lymphocytes are mainly involved in the subsequent inflammatory response, gradually forming pleural granulomas [3–5]. Tuberculous pleurisy is easily missed and misdiagnosed due to its insidious onset, slow course, and lack of specificity in diagnostic methods; therefore, tuberculous pleurisy needs to be diagnosed by multiple modalities.

Patients with tuberculous pleurisy usually have an acute or subacute onset, with 75% of patients presenting with chest pain, 70% with cough, 85% with night sweats, 50% with dyspnea, and 25% to 85% with weight loss [5, 6]. Complications of tuberculous pleurisy include tuberculous pneumothorax (purulent effusion caused by chronic active tuberculous pleurisy infection with a large collection of neutrophils), pleural thickening, celiac disease, and effusion pneumothorax (tuberculous pleural effusion caused by cavitary pulmonary tuberculosis that develops into a pneumothorax after drainage of the effusion).

The diagnostic value of routine examination of pleural effusion for tuberculous pleurisy consists in the following: for the diagnosis of pleural effusion, it should first be determined whether it is leaking or exuding fluid. The criteria for determining exudate [7] are as follows: (i) the ratio of pleural effusion to total serum protein is >0.5; (ii) the level of lactate dehydrogenase (LDH) in pleural effusion is >200 U/L; and (iii) the ratio of pleural effusion to serum LDH is >0.6. Tuberculous pleural effusion is exudate, and in addition to the characteristics of exudate, its appearance is usually colorless. Tuberculous pleural effusion is an exudate that, in addition to having exudative features, is usually colorless or straw (yellowish) in appearance and can also be turbid or bloody. The glucose content of tuberculous pleural fluid is significantly lower than that of blood glucose, and cytologic examination reveals a polymorphic pattern of cells in the pleural fluid [8], predominantly lymphocytes. In indeterminate cases, invasive tests are required to clarify the diagnosis, as shown in Figure 1.

The following methods have been studied for the diagnostic value of pathogenesis in tuberculous pleural effusions. With the advent of automated fluid culture systems, *Mycobacterium tuberculosis* has been cultured from pleural fluid and pleural tissue in up to 70% of cases [9]. Waldo [9] reported that the sensitivity of fluid culture of pleural fluid could reach 63% and that the time to report positive fluid culture was only 18 d [10]. In order to find the diagnostic value of pathogenesis in tuberculous pleural effusions, the following methods were presented.

With the development of science and technology, the diagnostic process in tuberculous pleural effusion has become more and more complex. It has been a great challenge to build the system model of the controlled object directly through the system identification method [6]. Many scholars have started to focus on the research of data-driven control algorithms. The model-free adaptive iterative learning control (MFAILC) is a typical data-driven control algorithm [7]. The method achieves model-free iterative learning control of an unknown nonlinear system by building a dynamic linearized data model equivalent to the nonlinear system along the iteration axis using compact-form dynamics linearization (CFDL) at each operating point and estimating the parameters in the model online using the input and output data of the controlled system. Model adaptive and interactive learning control of unknown nonlinear systems have been reported [6–8]. In the diagnostic application of tuberculous pleural effusion, due to the limited processing speed, memory capacity, and communication bandwidth of the IPC, an event-triggered control mechanism was proposed [11]. In this mechanism, only the trigger moment is used for computing and information transfer, which effectively reduces the number of controls and communication burden.

In order to facilitate clinicians to diagnose patients with tuberculous pleurisy at an early stage, help patients to obtain treatment early, and reduce lung damage, it is hoped that new techniques will be available in the future to help clinicians diagnose tuberculous pleurisy quickly. To address this issue, in this paper, we are going to investigate the problem of bidirectional consistency based on event-triggered iterative learning. First, a dynamic linearized data model of TB pleurisy intelligent system is established by using compact-form dynamic linearization method, and a parameter estimation algorithm of TB pleurisy data model is proposed; then, based on this data model, an output observer and a dead zone controller are designed, and an event-triggered distributed model-free iterative learning bidirectional consistency control strategy is constructed by combining with signal graph theory.

In the subsequent section, the proposed model iteration scheme is presented where the concept of the algebraic graph theory is explained. In Section 3, various results, which are collected or achieved during the experimental setup, are presented along with comparison with other existing state-of-the-art scheme. Furthermore, a brief discussion on how the problem is identified and effectiveness of the proposed system is described in detail. Finally, concluding remarks are given.

## 2. Model Iteration Scheme

### 2.1. Algebraic Graph Theory

In this paper, the communication topology of tuberculous pleural effusion diagnosis system is expressed as $\bar{𝒢}\;=\left(\bar{𝒱},\bar{ℰ},𝒜\right)$, in which $\bar{𝒱}=𝒱\cup \left\{0\right\},\;\bar{ℰ}\subseteq \bar{𝒱}\times \bar{𝒱}\cdot 𝒜=\left[a_{ij}\right]\in R^{N\times N},\;𝒱=\left\{1,2,\ldots ,N\right\}$), and *ℰ*⊆{(*i*, *j*)*|i*, *j* ∈ *𝒱*}⊆*𝒱* × *𝒱* represent the adjacency matrix of Fig $\bar{𝒢}$, vertex set, and edge set respectively, and *a*_*ij*_ ∈ {−1,0,1} is the weight value. The elements (*I*, *J*) in *ℰ* represent an edge between agents *I* and *J*, and the signal can be transmitted from agent *I* to agent *J*. At this time, if the relationship between agents *I* and *J* is cooperative, then *a*_*ij*_=1. In case of competitive relationship, *a*_*ij*_=−1.

In addition, when (*i*, *j*) ∉ *ℰ*, *a*_*ij*_=0. The adjacent agent set of agent *I* is *N*_*i*_={*j* ∈ *𝒱|*(*j*, *i*) ∈ *ℰ*}, and its penetration is *d*_*i*_=∑_*j*=1_^*N*^|*a*_*ij*_|, and the penetration of each agent constitutes the degree matrix *𝒟*=diag(*d*_1_, *d*_2_,…, *d*_*N*_) of figure $\bar{𝒢}$. The Laplace matrix of figure is ℒ=*𝒟* − *A*. In this paper, all nodes are divided into sets *𝒱*_1_ and *𝒱*_2_, of which *𝒱*=*𝒱*_1_ ∪ *𝒱*_2_ and *𝒱*_1_∩*𝒱*_2_=*ϕ*, *𝒱*_2_=*ϕ*. If agents *I* and *J* belong to the same set, they are cooperative relations; otherwise, it is a competitive relationship. In addition, matrix ℬ=diag(*b*_1_, *b*_2_,…, *b*_*N*_) is used to represent the connection relationship between the virtual leader and all followers. If agent *I* is directly connected with the virtual leader, then *b*_*i*_ = 1; otherwise *b*_*i*_ = 0.

### 2.2. Model Description

A class of SISO (single-input single-output) nonlinear, discrete-time tuberculous pleural effusion diagnosis system with one virtual leader and *N* followers is considered, in which the dynamic model of agent *I* satisfies the following equivalent form:

(1) $$\begin{array}{c} y_{i}\left(l,k+1\right)=f_{i}\left(y_{i}\left(l,k\right),\ldots ,y_{i}\left(l,k-n_{y}\right)u_{i}\left(l,k\right),\ldots ,u_{i}\left(l,k-n_{u}\right)\right), \end{array}$$

where *u*_*i*_(*l*, *k*) ∈ *R*, *y*_*i*_(*l*, *k*) ∈ *R* represent the input and output of agent *I* = 1, 2,…, *n*, respectively, *l* = 1, 2,…, *n* is the number of iterative steps, *K* ∈ {0, 1,…, *t*} is the time interval, *n*_*y*_ ∈ *R* and *n*_*u*_ ∈ *R* are unknown positive integers, and *f*_*i*_(.) is unknown nonlinear function. In addition, *y*_0_(*l*, *k*) is defined as the output of the virtual leader, which is represented by vertex 0 in the topology diagram $\bar{𝒢}$.

*Proposition 1* [1, 2]. *f*_*i*_(.) is a continuous nonlinear function with partial derivatives of.

*Proposition 2* [5, 12]. Equation (1) satisfies the generalized Lipschitz continuity condition along the iterative axis; that is, there is a constant *R* such that Δ*y*_*i*_(*l*, *k*+1)=Γ_*i*_(*l*, *k*)Δ*u*_*i*_(*l*, *k*)|Δ*y*_*i*_(*l*, *k*+1)| ≤ *r*|Δ*u*_*i*_(*l*, *k*)|, where Δ*y*_*i*_(*l*, *k*+1)=*y*_*i*_(*l*, *k*+1) − *y*_*i*_(*l* − 1, *k*+1), Δ*u*_*i*_(*l*, *k*)=*u*_*i*_(*l*, *k*) − *u*_*i*_(*l* − 1, *k*), and |Δ*u*_*i*_(*l*, *k*)| < *a*, are normal numbers. *Lemma 1* [5]. If equation (1) satisfies assumptions 1 and 2, equation (1) can be expressed by the following compact dynamic linearization model:

(2) $$\begin{array}{c} \Delta y_{i}\left(l,k+1\right)=\Gamma_{i}\left(l,k\right)\Delta u_{i}\left(l,k\right), \end{array}$$

where Γ_*i*_(*l*, *k*) ≤ *r* is a normal number, Γ_*i*_(*l*, *k*) is called pseudopartial derivative and is time-varying.

*Proposition 3*. Γ_*i*_(*l*, *k*) > 0 or Γ_*i*_(*l*, *k*) < 0 in equation (2). In this paper, as in literature [5], suppose Γ_*i*_(*l*, *k*) < 0.

The local error of distributed bidirectional consistency is defined as follows:

(3) $$\begin{array}{c} \zeta_{i}\left(l,k\right)=\sum_{j\in N\left(i\right)}\left|a_{ij}\right|\left(\mathrm{sign}\left(a_{ij}\right){\hat{y}}_{j}\left(l,k\right)-{\hat{y}}_{i}\left(l,k\right)\right)+b_{i}\left(s_{i}y_{0}\left(l,k\right)-{\hat{y}}_{i}\left(l,k\right)\right). \end{array}$$

Among them, if the agent *I* can directly obtain the target trajectory information from the virtual leader 0, that is, $\left\{0,i\right\}\in \bar{\varepsilon }$, *b*_*i*_=1; otherwise, *b*_*i*_=0. In addition, ${\hat{y}}_{i}\left(l,k\right)$ is the estimation of *y*_*i*_(*l*, *k*). Let *e*_*i*_(*l*, *k*)=*s*_*i*_*y*_0_(*l*, *k*) − *y*_*i*_(*l*, *k*) represent the tracking error and define ${\hat{e}}_{i}\left(l,k\right)=s_{i}y_{0}\left(l,k\right)-{\hat{y}}_{i}\left(l,k\right)$ as the estimation error, where when *i* ∈ *v*_1_, *s*_*i*_=1; *s*_*i*_=−1 when *i* ∈ *v*_2_.

*Proposition 4*. There is a directed spanning tree in figure $\bar{𝒢}$, and the virtual leader is the root node of the directed spanning tree; that is, the trajectory information of the virtual leader can be transmitted to all followers directly or indirectly.

**Definition 1 .**

If and only if the outputs of agent *I* and virtual leader meet the following conditions, the tuberculous pleural effusion diagnosis system is said to achieve two-way (bounded) consistency:

(4) $$\begin{array}{c} \underset{l⟶\infty }{\lim}\left(y_{i}\left(l,k\right)-s_{i}y_{0}\left(l,k\right)\right)=\iota . \end{array}$$

Among them, *ι* is a very small normal number, *I* = 1, 2,…, *n*.

## 3. Data and Methods

### 3.1. Data Collection

112 patients with pleural effusion treated in our hospital from June 2018 to June 2019 were selected as the research object. According to the clinical diagnosis and treatment guidelines of tuberculous pleurisy of the Chinese Medical Association [2], 76 patients were with tuberculous pleural effusion (tuberculosis group) and 36 patients with nontuberculous pleural effusion (nontuberculosis group). There were 86 males and 30 females. The age was (59.02 ± 4.94) years. Before treatment, the pleural effusion T-SPOT.TB, peripheral blood T-SPOT.TB, pleural effusion Xpert MTB/RIF, and pleural effusion ADA of each patient were collected for detection, and the detection results were analyzed retrospectively.

### 3.2. Inspection Method

#### 3.2.1. Pleural Effusion T-SPOT.TB

The reagent is T-SPOT.TB (Oxford Immunotec Ltd). Before treatment, 80∼100 ml of pleural effusion was reserved, and a piece of heparin sodium (12500 IU) was added for anticoagulation. The samples were sent for examination in time to ensure the freshness of the samples. Antigen A, antigen B, negative control (nonserum medium), and positive control (phytohemagglutinin) were tested, respectively, and the test results were interpreted.

#### 3.2.2. Peripheral Blood T-SPOT.TB

T-SPOT.TB reagent (Oxford Immunotec Ltd, UK) was used to isolate peripheral blood monocytes in strict accordance with the product reagent instructions, count and adjust the cell concentration.

#### 3.2.3. T-SPOT.B

The positive judgment standard is as follows: when the number of negative control spots is 0∼6, (number of antigen A or antigen B spots) − (number of negative control spots) ≥ 6. When the number of negative control spots ≥6, (number of antigen A or antigen B spots) ≥2 times (number of negative control spots) [4].

#### 3.2.4. Pleural Effusion Xpert MTB/RIF

The Xpert MTB/RIF detector and kit produced by CEPH Eid company of the United States were used. Pleural effusion was routinely reserved. Digestive fluid was added to the sample. The ratio of digestive fluid to pleural effusion was 1 ∶ 1 (V/V). Tighten the test tube cover and shake repeatedly for several times. Place it at room temperature for 15 min. When there is no visible block in the specimen, extract 2 ml specimen, add it into Xpert MTB/RIF reaction kit, put it into gene Xpert platform, wait for 2 h, and check the detection results of tuberculosis.

#### 3.2.5. Detection of Adenosine Deaminase (ADA) in Pleural Effusion

Adenosine deaminase reagent (Zhejiang Yilikang Biological Technology Co., Ltd.) is used to take 5∼10 ml of pleural effusion from the patient, add it into anticoagulant glass test tube, and operate in strict accordance with the reagent instructions. ADA value >40 U/L is regarded as positive.

### 3.3. Data Results

#### 3.3.1. Comparison of Test Results of Four Methods

The test results of pleural effusion T-SPOT.TB, peripheral blood T-SPOT.TB, pleural effusion Xpert MTB/RIF, and pleural effusion ADA are shown in Table 1. Among the 76 patients with tuberculous pleural effusion, 74 cases were positive for T-SPOT.TB in pleural effusion, 58 cases were positive for T-SPOT.TB in peripheral blood, 50 cases were positive for Xpert MTB/RIF in pleural effusion, and 22 cases were positive for ADA in pleural effusion. Among the 36 patients with nontuberculous pleural effusion, 28 cases were negative for pleural effusion T-SPOT.TB, 20 cases were negative for peripheral blood T-SPOT.TB, 36 cases were negative for pleural effusion Xpert MTB/RIF, and 18 cases were negative for pleural effusion ADA. Compared with clinical diagnosis, the difference was statistically significant (*x*^2^ = 70.34, 11.07, 42.78, and 4.72, *P* < 0.05).

#### 3.3.2. Efficiency Analysis of Individual Detection

The sensitivity of pleural effusion T-SPOT.TB (97.37%) was significantly higher than that of peripheral blood T-SPOT.TB (76.32%), Xpert MTB/RIF (65.79%), and ADA (28.95%) (*x*^2^ = 14.74, 25.22, 76.45, *P* ＜ 0.01). The specificity of Xpert MTB/RIF in pleural effusion (100%) was significantly higher than that of T-SPOT.TB in pleural effusion (77.78%), T-SPOT.TB in peripheral blood (55.56%), and ADA in pleural effusion (50.00%) (*x*^2^ = 6.89, 20.57, 24.00, *P* ＜ 0.01).

If the pleural effusion Xpert MTB/RIF and pleural effusion T-SPOT.TB are positive, it is determined as positive, and if two of them are negative or one of them is negative, it is determined as negative. The sensitivity of pleural effusion Xpert MTB/RIF and pleural effusion T-SPOT.TB was 64.47%, which was lower than that of pleural effusion T-SPOT.TB alone (97.37%); the difference was statistically significant (*x*^2^ = 26.63, *P* < 0.01), but the specificity was increased from 77.78% of pleural effusion T-SPOT.TB to 100%; the difference was statistically significant (*x*^2^ = 45.82, *P* < 0.01). See Table 2.

### 3.4. Proposed Working Curve Analysis

In this paper, the receiver operating characteristic (ROC) curve was used to analyze the best boundary value for the diagnosis of tuberculous pleural effusion. The areas under the ROC curve (AUC) of pleural effusion T-SPOT.TB, peripheral blood T-SPOT.TB, and Xpert MTB/RIF pleural effusion ADA were 0.91, 0.66, 0.81, and 0.45, respectively. The detection efficiency of pleural effusion T-SPOT.TB was significantly higher than that of peripheral blood T-SPOT.TB, pleural effusion Xpert MTB/RIF, and pleural effusion ADA. See Figure 2.

## 4. Numerical Simulation and Analysis

This simulation experiment is mainly aimed at the application background that the injection direction of proportional valve in the upper cleaning area and filling area of tuberculous pleural effusion is opposite, and the two-way consistency simulation experiment of event-triggered model-free iterative learning is carried out.

The site of tuberculous pleural effusion is shown in Figure 3, in which the valve nozzle of proportional valve is shown, and the autoregressive model of this kind of proportional valve is identified as follows:

(5) $$\begin{array}{c} \frac{y_{i}\left(l,k+1\right)}{u_{i}\left(l,k\right)}=\frac{\left(1.24z^{-1}-0.93z^{-2}\right)}{\left(1-1.6z^{-1}+0.6z^{-2}\right)}, \end{array}$$

where *y*_*i*_(*l*, *k*) is the pressure at the nozzle and *u*_*i*_(*l*, *k*) is the opening of the proportional valve.

The target pressure value is defined as follows:

(6) $$\begin{array}{c} y_{0}\left(l,k\right)=0.5\;\sin\left(\frac{k\pi }{20}\right)+0.3\;\cos\left(\frac{k\pi }{10}\right). \end{array}$$

Here *k* ∈ [0,100],  *l* ∈ [0,400].

This experiment consists of a tuberculous pleural effusion diagnostic system with seven proportional valve control systems, in which the intelligences are grouped into two groups: *v*_1_ (1, 2, 7) and *v*_2_ (3, 4, 5, 6). The communication topology is shown in Figure 4, where 0 represents the virtual leader, black arrows represent the cooperative relationship, and red arrows represent the competitive relationship. According to the graph theory, the maximum value of diagonal elements in *L* + *B* is 2, so we can set *β* = 0.24, and the remaining parameter values are *λ* = 1, *χ* = −1.4, *u* = 0.55, *δ* = 0.5, *ρ* = 0.5, and *σ* = 10^−4^. The initial values are set as follows:

(7) $$\begin{array}{c} {\hat{\Gamma }}_{i}\left(1,k\right)=2,\\ u_{i}\left(0,0\right)=\mathrm{rand}\left(-0.005,0.005\right),\\ y_{i}\left(0,0\right)=\mathrm{rand}\left(-0.005,0.005\right),\\ i=1,2,3,4,5,6,7. \end{array}$$

The experimental results are shown in Figures 5–7, which show that the error is large at the beginning, but then the tracking error of the follower converges rapidly to near 0 with the increase of the iteration steps. From Figure 5, it can be seen that the trigger moments are intermittent, thus verifying that the designed dead zone controller effectively avoids the Zeno-like phenomenon of the trigger [13], where the trigger times of each intelligence are 30, 37, 27, 40, 44, 43, and 28, with an average trigger time of 35.57. Compared with the algorithms in papers [5–7, 12], the algorithm not only achieves bidirectional consistency tracking, but also reduces the communication resources by 64.43% so that the control protocol designed in this paper has better energy saving effect and control performance.

## 5. Discussion

Tuberculous pleural effusion accounts for 49.5% to 54.5% of patients with pleural effusion [5], and the positive rate of pleural effusion smear for *Mycobacterium* antacid is only 0% to 25%, and the positive rate of pleural effusion culture for *Mycobacterium tuberculosis* is 11.7% to 56.8% [6]. Therefore, there is a clinical need for a rapid and effective test for early diagnosis, early treatment, and reduction of complications such as pulmonary destruction due to tuberculous pleural effusion.

The peripheral blood T-SPOT.TB assay is an enzyme-linked immunospot technique that detects the number of interferon-releasing effector T cells from monocytes in peripheral blood samples stimulated by *Mycobacterium tuberculosis-* (MTB-) specific antigens, using the RD1 gene of MTB encoding a secreted antigen target (ESAT-6) with a relative molecular weight of 6,000 and culture filtration protein (CFP-10) with a relative molecular weight of 10,000 as specific antigens and culture filtration protein (CFP-10) with a relative molecular weight of 10,000 as specific antigens. This method is increasingly used in the diagnosis of clinical tuberculosis [12]. However, peripheral blood T-SPOT.TB has its own defects and is easily influenced by the number of T lymphocytes in peripheral blood [6], which often results in false-positive results. (1) The T-SPOT.TB test technique cannot distinguish between latent TB infection and active TB. (2) There are some special nontuberculous mycobacterial infections, such as *Mycobacterium marinum*\*Mycobacterium kansasii* infection; the T-SPOT.TB test may also sometimes show false positive results. (3) Presence of some extrapulmonary TB that is not currently detectable. (4) Infections, inflammation with concurrent transient infections, may also show positive T-SPOT.TB results [7]. (5) In some cancer patients, tumor antigens have cross-epitopes with two TB antigens (CFP-10, ESAT-6), resulting in immune responses of tumor T cells to both TB antigens, which limits the specificity of the diagnosis of active TB.

## 6. Conclusions

In order to facilitate clinicians to diagnose patients with tuberculous pleurisy early, help patients to get treatment early, and reduce lung damage, it is hoped that in the future new techniques can help clinicians to diagnose tuberculous pleurisy quickly. To this end, this paper investigates the bidirectional consistency problem based on event-triggered iterative learning, designs an output observer and a dead zone controller, and constructs an event-triggered distributed model-free iterative learning bidirectional consistency control strategy by combining signal graph theory. In this paper, we collect data from patients with pleural effusion. The experimental results showed that the differences between pleural effusion Xpert MTB/RIF (65.79%, 50/76) and pleural effusion ADA (28.95%, 22/76) were statistically significant (*x*^2^ = 14.74, 25.22, and 76.45, *P* < 0.01). Conclusively, the T-SPOT.TB test for pleural effusion has a high sensitivity and the Xpert MTB/RIF test for pleural effusion has a high specificity, and the combination of the two tests can significantly improve the specificity of the diagnosis of tuberculous pleural effusion, which is worthy of clinical promotion.

## Figures and Tables

**Figure 1:** Diagnostic CT diagram in tuberculous pleural effusion.

**Figure 2:** ROC curves of four detection methods.

**Figure 3:** Tuberculous pleural effusion site (a) and nozzle (b).

**Figure 4:** Communication topology of the diagnostic control system for tuberculous pleural effusion.

**Figure 5:** Two-way consistency tracking effect of tuberculous pleural effusion diagnosis control system. (a) 8th iteration. (b) 355th iteration.

**Figure 6:** Bidirectional consistency tracking error diagram of the tuberculous pleural effusion diagnosis control system.

**Figure 7:** Event-triggered moment diagram at the 355th iteration.

**Table 1:** Comparison of the results of two detection methods.

Tst method	Tuberculosis group (*n* = 76)		Nontuberculosis group (*n* = 76)		Total (*n* = 112)		*x* ^2^ value	*P* value
	Number of cases	Percentage	Number of cases	Percentage	Number of cases	Percentage		
Pleural effusion T-SPOT.TB							70.34	<0.01
Negative	74	97.37	8	22.22	82	72.21		
Negative	2	2.63	28	77.78	30	26.79		
Peripheral blood T-SPOT.TB							11.07	<0.01
Positive	58	76.32	16	44.44	74	66.07		
Negative	18	23.68	20	48.56	38	33.83		
Pleural effusion Xpert MTB/RF							42.78	<0.01
Positive	50	65.79	0	0.00	50	44.64		
Negative	26	30.21	36	100.00	82	55.36		
Pleural effusion ADA							4.72	<0.05
Positive	22	28.95	19	50.00	40	35.71		
Negative	54	71.05	18	50.00	72	64.29		

**Table 2:** Comparison of pleural effusion Xpert MTB/RIF combined with pleural effusion T-SPOT test and four separate tests (%) (cases).

Tst method	Sensitivity	Specificity	Positive expected value	Negative expected value
Pleural effusion T-SPOT.TB	97.37 (74/76)	77.78 (28/36)	90.24 (74/82)	93.33 (28/30)
Peripheral blood T-SPOT.TB	76.32 (58/76)	55.56 (20/36)	78.39 (58/74)	52.63 (20/38)
Pleural effusion B/Rif	65.79 (50/76)	100.00 (36/36)	100.00 (50/50)	58.06 (36/62)
Pleural effusion ADA	28.95 (22/76)	50.00 (18/36)	55.00 (22/40)	25.00 (18/72)
Pleural effusion tot combined with pleural effusion Xpert TB/Rif	64.47 (49/76)	100.00 (36/36)	100.00 (49/49)	75.00 (36/18)

## Data Availability

The datasets used and analyzed during the current study are available from the corresponding author upon reasonable request.
